This article has been retracted.

# ARHGAP24 inhibits cell cycle progression, induces apoptosis and suppresses invasion in renal cell carcinoma

**DOI:** 10.18632/oncotarget.10386

**Published:** 2016-07-02

**Authors:** Gaosi Xu, Xiongbing Lu, Tianlun Huang, Jie Fan

**Affiliations:** ^1^ Department of Nephrology, The Second Affiliated Hospital of Nanchang University, Nanchang, China; ^2^ Department of Urology, The Second Affiliated Hospital of Nanchang University, Nanchang, China

**Keywords:** renal cancer, ARHGAP24, proliferation, cell cycle, apoptosis

## Abstract

Renal cell carcinoma (RCC) is the major cause of kidney malignancy-related deaths. Rho GTPases are key regulators in cancer cell metastasis. ARHGAP24, a Rac-specific member of the Rho GTPase-activating protein family, acts as a functional target of cancer cell migration and invasion. In the present study, we identified ARHGAP24 expression is downregulated in renal cancer tissues and is highly correlated with long-term survival in RCC patients. Therefore, we investigated the biological functions of ARHGAP24 in renal cancer cells. Ectopic expression of ARHGAP24 resulted in inhibited cell proliferation and arrested cell cycle in two renal cancer cell lines (786-0 and Caki-2); the results were confirmed by ARHGAP24 knocking down. In addition, ARHGAP24 significantly reduced the cell invasion ability and induced apoptosis in renal cancer cells. In addition, overexpressing ARHGAP24 impaired tumor formation *in vivo*. In summary, our results illustrated that ARHGAP24 plays a unique role in RCC progression as a tumor repressor.

## INTRODUCTION

Renal cell carcinoma (RCC) has the highest death rate among solid urological tumors [1, 2]. It has been reported that the number of patients with RCC has been increasing at a continuous and rapid rate recently [3, 4]. This tumor has become the 10th most common in men and the 14th most common in women [5].

Diagnostic technology has revolutionized in recent years, thus RCC patients have been diagnosed at the early stages, which enables the appropriate clinical interventions in time. Therapeutic treatment for early RCC, including surgical approaches, has improved RCC prognosis. However, RCC patients are generally resistant to chemotherapy, radiotherapy, and hormone therapy [6–8]. Therefore, to effectively control growth of cancer cells in RCC, especially in advanced stages, is a significant challenge. One of the reasons is that RCC pathogenesis and progression are not well defined [9]. The accumulating evidence on RCC using genetic approaches has indicated that many genes are unique in RCC [5, 10]. Therefore, a better understanding of the molecular mechanism in RCC metastasis will improve diagnostic classification and shed light on therapeutic approaches.

Rho family GTPases are key regulators of actin dynamics that contribute to many cellular processes including cell adhesion, migration, and differentiation [11, 12]. Many studies reported that abnormalities in Rho GTPases signaling result in development defects, immune response deficiency and cancer metastasis [13]. Rho GTPases cycle between GTP-bound (active) and GDP-bound (inactive). GTPase-activating proteins (GAPs) catalyze GTP hydrolysis to inactivate small GTPases [14]. ARHGAP family genes (ARHGAP24, ARHGAP22 and ARHGAP25) are members of Rho GAPs [15, 16]. ARHGAP24 (also known as FilGAP) is a Rac1 specific GAP. ARHGAP24 transcript is enriched in kidney tissues [17]. ARHGAP24 is a highly conserved gene and it is upregulated during podocyte differentiation *in vivo*, suggesting a potential role in kidney development [18]. The roles of ARHGAP24 in RCC progression remain largely unknown.

In the current study, we demonstrated that overexpressing ARHGAP24 decreases cell proliferation, slows cell cycle progression, increases apoptosis and inhibits metastasis. The roles of ARHGAP24 were confirmed using ARHGAP24 siRNA. The GSEA dataset confirmed that cell cycle and apoptosis signaling pathways are correlated with ARHGAP24 expression.

## RESULTS

### Decreased expression of ARHGAP24 in RCC tumor tissues

To define ARHGAP24 expression patterns in RCC, we first examined mRNA levels of ARHGAP24 in 80 patients diagnosed with RCC. Tumor tissues were compared with adjacent unaffected tissues from the same patient. We found that ARHGAP24 mRNA is dramatically decreased in renal tumor tissues (Figure 1A). Similar results were obtained after analyzing a TCGA dataset (Figure 1B). To investigate whether similar changes at translation level, we performed immunohistochemistry staining. ARHGAP24 is abundant in normal tissues and the expression is significantly reduced in tumor tissues both at transcription and translation levels (Figure 1C). ARHGAP24 was absent in 60.9% patients (128 out of 210).

**Figure 1:** High expression of ARHGAP24 indicates better survival of renal cancer **A.** The expression level of ARHGAP24 in 80 patients' renal tumor tissues and adjacent tissues. **B.** ARHGAP24 expression was significantly decreased in renal tumor tissues when compared with the adjacent tissues based on the data from the TCGA dataset (*p*<0.0001). **C.** Upper panel: immunostaining of ARHGAP24 in renal cancer and unaffected tissues. Scale bar: 100 μm. Lower panel: representative ARHGAP24 protein expression in renal cancer (T1, T2, T3 and T4) and unaffected tissues (N1, N2, N3 ad N4). **D.** Survival analysis of 70 patients with renal cancer. **E.** Survival analysis of patients from the TCGA KIRC dataset. The survival time in ARHGAP24 high expression patients was notably longer than patients with low ARHGAP24 expression.

Next, to evaluate whether there is correlation between ARHGAP24 protein expression and clinicopathological characteristics in RCC patients, we performed a Chi-square test. Low ARHGAP24 expression is correlated with tumor extent, lymph node metastasis, distant metastasis and Fuhrman grade (Table 1). Furthermore, univariate analysis identified that ARHGAP24 expression is negatively correlated with several prognostic factors: tumor extent (*P*<0.01), lymph node metastasis (*P*<0.05), distant metastasis (*P*<0.01) and Fuhrman grade (*P*<0.05) (Table 2). Interestingly, multivariate analysis demonstrated that ARHGAP24 expression, tumor extent, lymph node metastasis and distant metastasis are independent prognostic factors for RCC mortality (Table 2).

**Table 1:** Correlations between ARHGAP24 expression and clinicopathological features in patients with RCC (n=210)

ARHGAP24 expression				
General Characteristics	Total Number	Positive (n=82)	Negative (n=128)	*P* value
Age (years)				
< 65	126	45	81	0.2497
>=65	84	37	47	
Gender				
Male	124	48	76	1.000
Female	86	34	52	
Tumor extent (TNM 2009)				
pT1	121	50	71	0.0161*
pT2	45	23	22	
pT3	39	7	32	
pT4	5	2	3	
Regional lymph node metastasis (TNM 2009)				
N0	193	80	113	0.0183*
N1	17	2	15	
Distant metastasis (TNM 2009)				
M0	186	78	108	0.0244*
M1	24	4	20	
Fuhrman Grade				
I-II	159	69	90	0.0314*
III	51	13	38	

**Table 2:** Cox regression analysis of ARHGAP24 expression with cancer-specific mortality in renal carcinoma

	Univariate analysis		Multivariate analysis	
	HR (95% CI)	*P* value	HR (95% CI)	*P* value
ARHGAP24 (high/low)	0.113(0.064-0200)	0.000***	0.0507 (0.0239-0.107)	0.000***
Age	0.862 (0.538-1.382)	0.537		
Gender	1.282 (0.808-2.034)	0.292		
Tumor extent	1.434(1.119-1.837)	0.004**	1.438 (1.057-1.956)	0.021*
Regional lymph node metastasis	2.087 (1.037-4.200)	0.039*	6.967 (2.794-17.374)	0.000***
Distant metastasis	3.537 (2.047-6.111)	0.000***	2.123 (1.123-4.012)	0.020*
Fuhrman Grade	1.794(1.101-2.925)	0.019*	1.499 (0.843-2.663)	0.168

Kaplan-Meier analysis of our patient data and TCGA dataset showed that the overall survival time of higher-ARHGAP24-expressing individuals is notably longer than the lower-ARHGAP24-expressing individuals (Figure 1D, 1E). These results suggested that down-regulation of ARHGAP24 expression in renal cancer patients contributes to poor survival. ARHGAP24 may serve a potential biomarker for predicting RCC prognosis. Next, to further understand the clinical significance of the above findings, we studied the biological roles of ARHGAP24 in renal cancer cell lines.

### Effects of ARHGAP24 on cell viability in renal cell lines

First, we compared the expression level of ARHGAP24 in 5 renal cancer cell lines (786-0, ACHN, Caki-1, Caki-2 and A498) using real-time PCR and western blot. 786-0 and Caki-2 exhibited lower levels of ARHGAP24 in both mRNA and protein expression (Figure 2A, 2B). Interestingly, ARHGAP24 expresses in a comparable level in HK-2 proximal tubule cell line (Figure 2A, 2B). Since we noticed that a high ARHGAP24 expression level associates with increased patient survival, we sought to explore the hypothesis that ARHGAP24 is a tumor suppressor in RCC progression. We used 786-0 and Caki-2 cell lines in the following study because of the low ARHGAP24 expression at the baseline. We overexpressed ARHGAP24 in 786-0 and Caki-2 using viral infection (Figure 2C, 2D). Overexpressing ARHGAP24 resulted in a decreased cell growth rate at 24, 48 and 72 h in both 786-0 and Caki-2 cells (Figure 2F, 2G). We applied ARHGAP24 siRNA in ACHN cells because the endogenous ARHGAP24 levels are abundant (Figure 2A, 2B). Knocking down ARHGAP24 in ACHN cells promoted cell growth (Figure 2H). These results suggested that ARHGAP24 serves as an inhibitory regulator in renal cancer cell proliferation.

**Figure 2:** ARHGAP24 inhibits cell growth of renal cancer cells **A.** mRNA levels of ARHGAP24 in 5 renal cancer cell lines and HK-2 cells. **B.** Protein expression of ARHGAP24 in 5 renal cancer cell lines and HK-2 cells. **C, D.** Overexpression of ARHGAP24 in 786-0 and Caki-2 cells. **E.** Knockdown of ARHGAP24 expression in ACHN cells. **F, G.** Cell proliferation was detected at 12, 24, 48 and 72 h after transfection in 786-0 and Caki-2 cells. **H.** Knocking down ARHGAP24 promoted cell proliferation in ACHN cells. Three independent experiments were performed, and data were represented as mean ± SD, ^**^P<0.01.

### ARHGAP24 promotes G1/S cell cycle progression and increases apoptosis in renal cancer cells

Next, we explored the mechanisms of ARHGAP24's inhibitory effects in proliferation. First, we performed GSEA analysis on a KEGG dataset, and we found that cell cycle and apoptosis pathway makers are strongly associated with ARHGAP24 high expression (Figure 3A).

**Figure 3:** ARHGAP24 promotes G1/S phase transition **A.** Cell cycle and apoptosis analysis and ARHGAP24 expression. **B, C, D.** Cell cycle was analyzed using flow cytometry in ARHGAP24 overexpressing cells in 786-0 cells (B) and Caki-2 cells (C), or ARHGAP24 siRNA in ACHN cells (D). **E, F.** Cell cycle proteins PCNA, CDK1 and CDK2 were altered with ARHGAP24 levels. *P<0.05; **P<0.01. Three independent experiments were performed, and data were represented as mean ±SD.

We then examined the effects of ARHGAP24 on cell cycle in 786-0 and Caki-2 cells. Flow cytometry analysis revealed that cells infected with ARHGAP24 exhibit a significant increase in G0/G1 phase proportion, and a decrease in S phase percent compared to mock cells (Figure 3B, 3C). Consistent with overexpression, ARHGAP24 siRNA in ACHN cells efficiently decreased G0/G1 and increased S phase proportion (Figure 3D). Furthermore, we used western blot to evaluate three cell cycle regulating proteins: PCNA, CDK1 and CDK2. We found that PCNA, CDK1 and CDK2 are significantly down-regulated by the overexpressing of ARHGAP24 in both cell lines (Figure 3E, 3F). Together, these results suggested that ARHGAP24 has anti-proliferative effects on renal cancer cells.

To evaluate the apoptotic function of ARHGAP24, we performed an Annexin V-FITC/PI staining assay. As shown in Figure 4A and 4B, overexpressing ARHGAP24 in renal cancer cells significantly induced cell apoptosis. Consistent with ARHGAP24 overexpression, knocking-down ARHGAP24 using siRNA reduced cell apoptosis (Figure 4C). We compared protein levels of two apoptotic promoting proteins (Bax and Casepase3) and an anti-apoptotic protein (Bcl-2) by western blot. We found that the Bax and Casepase3 proteins are up-regulated by overexpressing ARHGAP24, whereas Bcl-2 is down-regulated (Figure 4D, 4E).

**Figure 4:** ARHGAP24 promotes cell apoptosis in renal cancer cells **A, B, C.** ARHGAP24 was overexpressed in 786-0 and Caki-2 cells or knocked down in ACHN cells. (C) 786-0 (A), Caki-2 (B) and ACHN cells (C) were stained with annexin V-flurescein and apoptosis rates were examined using flow cytometry. **D, E.** Aspoptotic factors Bax, Caspase3 and Bcl-2 were altered after overexpressing ARHGAP24. **P<0.01. Three independent experiments were performed, and data were represented as mean ±SD.

### ARHGAP24 decreases metastasis in renal cancer cells

Metastasis is another essential behavior of cancer cells. We wondered whether ARHGAP24 regulates metastasis in renal cancer cells. 786-0 and Caki-2 cells were transfected with ARHGAP24, ACHN cells were transfected with ARHGAP24 siRNA, and the cell invasion was evaluated by *in vitro* invasion assay. ARHGAP24 overexpressing cells showed significantly reduced invasion capability compared to the MOCK group (Figure 5A, 5B). Consistent with this, ARHGAP24 knock-down in ACHN cells significantly enhanced cell invasion (Figure 5C). These results suggest that ARHGAP24 inhibits cell invasive behavior.

**Figure 5:** ARHGAP24 decreases cell invasion in renal cancer cells **A.** Overexpression of ARHGAP24 in 786-0 notably inhibited cell invasion (^**^P<0.01). **B.** Overexpression of ARHGAP24 in Caki-2 cells significantly inhibited cell invasion (^**^P<0.01). Three independent experiments were performed, and data were represented as mean ±SD. **C.** Knocking down ARHGAP24 in ACHN significantly promoted cell invasion (**P<0.01). Scale bar: 100 μm (A, B), 50 μm (C).

### ARHGAP24 inhibits RCC growth in the nude mice xenograft model

Finally, we examined whether overexpressing ARHGAP24 could reduce tumor growth *in vivo*. Caki-2 cells, infected with mock plasmid (as control) or ARHGAP24, were subcutaneously injected in nude mice; and tumors were measured on day 46 after injection. Tumors in the ARHGAP24 overexpressing group grew slower than the control group. Tumor weight was significantly decreased in the ARHGAP24 group (Figure 6). These data suggested that overexpression of ARHGAP24 inhibits tumor growth in nude mice. These *in vivo* data strengthened and confirmed our *in vitro* results that ARHGAP24 contributes to RCC tumorgenesis, as a tumor suppressor.

**Figure 6:** Over-expression of ARHGAP24 in renal cancer cells reduces tumor growth *in vivo* **A.** Caki-2 cells transfected with either ARHGAP24 or control vector (MOCK) were subcutaneously injected in athymic nude mice. Tumor volume was evaluated for 18-48 days. **B.** At day 46, mice were sacrificed and tumors were examined. Tumor growth was significantly reduced in the ARHGAP24 overexpression group.

## DISCUSSION

In the current study, we investigated the biological function of ARGHP24 in RCC progression. The clinical analysis illustrated that ARHGAP24 is significantly decreased in patients with RCC, which was confirmed by the TCGA dataset. Overexpression of ARHGAP24 in renal cancer cells inhibited cell growth and invasion, and induced cell apoptosis. We characterized for the first time that ARHGAP24, a member of ARHGAP family genes, is downregulated in renal cancer tissue and exhibits anti-tumor and cytotoxic effects in renal cancer cells.

Rho GTPases are key regulators in cytoskeleton dynamics, and therefore control different steps of cell migration, focal adhesion and cell cycle progression [19], which are key cancer cell behaviors. Small GTPases cycle between an active GTP-bound state and an inactive GDP-bound state. GAPs promote the transition from GTP to GDP [20, 21]. Although several GAPs have been indicated as major regulators in multiple cancers [22, 23], the mechanisms underlying GAPs are understudied. ARHGAP24 (also known as FilGAP) is expressed ubiquitously in majority of tissues, with the highest expression level in kidney [17], suggesting an essential role in renal cell development. Bioinformatics studies determined ARHGAP family (including ARHGAP24) is cancer-associated genes [24, 25], because their genetic alterations lead to carcinogenesis [26]. In particular, ARHGAP24 is an independent prognostic factor of malignant lymphomas [27]. ARHGAP24 is involved in breast cancer cell invasion and migration [28, 29], and it antagonizes mesenchymal invasion [30].

Although ARHGAP24 has been previously reported in regulating cell invasion and motility in multiple cancers, whether ARHGAP24 modulates RCC development remains unexplored. In this study, we demonstrated the relationship between the expression level of ARHGAP24 and clinical characteristics, as well as patient's prognosis from more than 200 individuals. There was no correlation between ARHGAP24 expression level and age or gender; but high expression of ARHGAP24 was associated with tumor extent, lymph node metastasis, distant metastasis and Fuhrman grade. These results indicate that ARHGAP24 is a tumor suppresser in renal cancer.

With the advance of tumor treatment, tumor suppressor genes and their biological functions serve as an important research focus. In RCC, the most representative tumor suppressor gene is VHL, which is known to inhibit tumor progression through various mechanisms, such as Wnt/β-catenin and HIF pathways. [31, 32]. We examined the effects of ARHGAP24 on proliferation, cell cycle and apoptosis using 786-0 and Caki-2 renal cancer cells. Overexpression of ARHGAP24 cells significantly reduces cell growth rate and promotes cell apoptosis. Moreover, cell cycle analysis showed that ARHGAP24 arrests G1/S cell cycle transition in renal cells. Further, overexpression of ARHGAP24 in 786-0 and Caki-2 cells significantly decreases tumor cell invasion capability. Interestingly, other studies found that silencing ARHGAP24 impaired breast cancer cell invasion and high ARHGAP24 causes maintenance of amoeboid features of lymphoma [27, 28]. It is possible that the interaction between ARHGAP24 and other molecules is context dependent and function through different molecular pathways in various types of cancer. For instance, the spatial and temporal activation of Rac (ARHGAP24 effector) could be one of the major determinants of cancer cell behaviors.

Despite the advances in technology, metastasis in cancer progression remains the leading challenge in cancer research. RCC is a malignant tumor in urinary systems, and the only effective therapeutic strategy is surgery for early diagnostic RCC patients at present. If metastasis occurs in RCC patients, the five-year survival rate is less than 10% [33]. It is critical to understand the cellular changes during the occurrence, development and metastasis of RCC. A better understanding of the molecular mechanisms of tumor suppressors will shed light on early diagnosis and provide future therapeutic strategies. Our clinical characterization of ARHGAP24 downregulation in RCC tissues suggests that ARHGAP24 is a potential tumor suppressor that is silenced during RCC development. Since new therapeutic target is urgently needed in RCC to combat cancer invasion, a further identification and analysis of ARHGAP24 biological functions in RCC will be conducted with the rationale that altered Rho GTPase signaling contributes to RCC progression and metastasis. In summary, as a tumor suppressor gene in RCC, ARHGAP24 serves as a useful prognosis marker and a potential target for the treatment of RCC in future.

Our study provided key evidences that suggest ARHGAP24 plays an essential role in proliferation, apoptosis and metastasis of renal cancer cells, as well as cell cycle progression and apoptosis. Since ARHGAP24 expression level is associated with tumor maximum diameter, patients' survival rate and renal metastasis, inhibition of ARHGAP24 might serve as a therapeutic strategy for RCC patients. Future studies will focus on the downstream signaling pathway of ARHGAP24 and the molecular mechanism of its tumor suppressor role in RCC.

## MATERIALS AND METHODS

### Patients and tissue samples

A total of 210 patients with RCC were chosen from the Second Affiliated Hospital of Nanchang University between January 2009 and June 2010. Clinical and pathological follow-up information was collected from all patients. Adjacent normal renal tissues served as the negative control in each case. Normal renal tissues were collected within 5 cm of tumor margin during surgical procedures. Ethical approval was provided by the independent ethics committee in the Second Affiliated Hospital of Nanchang University. Written consent was obtained from all patients, or their guardians, according to ethics committee guidelines.

### Immunohistochemistry

Tissues were fixed in 10% formaldehyde, embedded in paraffin, and were sectioned into 4μm slices. The slices were hydrated in 70% ethanol and washed with PBS. Antigen retrieval was conducted by heating slides for 5 minutes in a microwave in a 0.1 M citrate buffer (pH 6.0). Blocking was performed using endogenous peroxide with 3% H_2_O_2_ in methanol for 10 minutes. Sections were incubated with an antibody against ARHGAP24 (Abcam) for 1 hour, and then were incubated with biotin-labeled secondary antibodies for 30 min at room temperature. Signals were visualized by the ABC kit and DAB substrate (Vector Laboratory), and hematoxylin was used for nuclear staining.

### Cell lines and cell culture

Human renal carcinoma cell lines (786-0, ACHN, Caki-1, Caki-2 and A498), HK-2 human renal proximal tubule cells and HEK293 cells were purchased from the cell bank the Shanghai Branch of the Chinese Academy of Sciences (Shanghai, China). 293T cells were provided by the Shanghai Tumor Research Institute. Cells were grown in an DMEM medium with 10% fetal bovine serum (FBS) in the presence of penicillin/streptomycin at 37°C with 5% CO_2_.

### Plasmids

Lentiviral constructs of human ARHGAP24 (JRDUN Biotechnology, Shanghai) or mock plasmid were introduced into HEK293 cells to produce lentivirus. 786-0 and Caki-2 cells were infected with lentivirus and 48 hours after infection, cells were harvested for various assays.

Three ARHGAP24 siRNAs were designed (1 GGAGGAUACUGUUCGUUAU, 2 GCCAGGCUAAUCUUGUUAA, and 3 GAGUUUGCCAGUGGUAAAU). 3 was the most efficient one, thus #3 siRNA experiments were performed in ACHN cells.

### Reverse transcription and real-time PCR

Total RNA was extracted using Trizol. Quantitative real-time PCR was performed using SYBR Green PCR kits (Takara, Japan). The following primers were used: ARHGAP24 forward 5′-AACTCCTGTCGCTCTTCTACC-3′ and reverse 5′-GCTGTTGCCCACAAATGTCTC-3′, GADPH forward 5′-CACCCACTCCTCCACCTTTG-3′ and reverse 5′-CACCCACTCCTCCACCTTTG-3′. Gene expression was normalized to GADPH.

### Cell proliferation assay

Cell viability was examined using a Cell Counting Kit (CCK)-8 (Beyotime, Shanghai, China). Briefly, 4 × 10^3^ cells were seeded in a 96-well plate, and cells were harvested at 24, 48 and 72 hours, respectively. A CCK-8 reagent was added to each well 1 hour prior to harvest. The optical density (OD) of 450 nm was determined using a spectrophotometer. Triplicates were performed at each of the time points.

### Flow cytometry

For cell cycle analysis, cells were harvested at 48 hours and incubated with 50 μg/ml of propidium iodide (PI). Cell-cycle analysis was performed using flow cytometry (FACSCalibur, BD Biosciences). Cell apoptosis assay was performed using an Annexin V-APC/PI apoptosis detection kit. Apoptosis was analyzed using the same machine.

### Cell invasion assay

1×10^5^ cells were seeded in the upper chamber of 24-well Matrigel-coated invasion chambers. The chemotaxis gradient was set up by adding 10% DMEM medium to the lower chamber. After 48 hours, cells that had migrated to the lower chamber were fixed with formaldehyde, stained and counted.

### Western blot analysis

786-0 and Caki-2 cells were washed twice with PBS, and were collected in a lysis buffer. Membranes were blocked with 5% skim milk, followed by incubation with antibodies against ARHGAP24, Casepase3, PCNA, CDK1, CDK2 (Abcam, Cambrige, MA), Bax, Bcl-2(Santa Cruz, CA, USA) and GADPH (CST, Beverly, USA). After incubating with secondary antibodies, the signals were visualized using enhanced chemiluminescence (ECL, Millipore).

### Nude mouse xenograft experiments

Nude-mouse injection was performed by injecting Caki-2 cells. Tumor growth size was measured (length, height and width) every 3-4 days after tumor formation (around 1-2 weeks) as previously described [34]. Mice were sacrificed at 46 days after the injection, and the tumors were weighed.

### Statistical analysis

All data were presented as the mean ± SD. T tests were performed; survival time without RCC and overall survival time were analyzed by the Kaplan-Meier survival curves and long-rank nonparametric test; and *P*< 0.05 was considered as statistically significant.
